This article has been retracted.

# Neonatal congenital mesoblastic nephroma that caused respiratory oncologic emergency early after birth: a case report

**DOI:** 10.1186/s12887-022-03210-8

**Published:** 2022-03-17

**Authors:** Hirotaka Kato, Yasuyuki Mitani, Taro Goda, Hiroki Yamaue

**Affiliations:** Second Department of Surgery, Wakayama Medical University Hospital, 811-1 Kimiidera Wakayama, Wakayama, 641-8509 Japan

**Keywords:** Congenital mesoblastic nephroma, Dyspnea, Neonate, Oncologic emergency

## Abstract

**Background:**

Congenital mesoblastic nephromas mainly present as asymptomatic abdominal masses, but some present hematuria, hypertension or hypercalcemia. Neonatal dyspnea in an early-birth neonate due to rapid tumor growth is reported here for the first time.

**Case presentation:**

A renal tumor and polyhydramnios were detected by ultrasonography of a male fetus at 32 weeks and 3 days of gestation. The mother had abdominal distension due to the polyhydramnios and signs of imminent premature birth. Amniocentesis was performed and the signs of imminent preterm birth subsided, but growth of the renal tumor was noted as a potential cause of respiratory dysfunction. Cesarean section was performed at 36 weeks and 2 days of gestation. His birthweight was 2638 g and his 1 and 5 min APGAR scores were 2 and 4 points, respectively. There was no spontaneous breathing at birth and he had remarkable abdominal distention. He underwent cardiopulmonary resuscitation. After circulation stabilized, emergency surgery was performed because of progressive hypoxemia and respiratory acidosis. Laparotomy revealed a huge tumor arising from the right kidney and right nephrectomy was performed. Histopathological examination led to diagnosis of congenital mesoblastic nephroma. The respiratory condition and circulatory dynamics stabilized after the pressure on the thorax from the tumor was relieved by surgery. The postoperative course was uneventful. No recurrence or complications have been observed in the 36 months since the surgery.

**Conclusions:**

Congenital mesoblastic nephroma can rapidly increase in size from the fetal period and may cause respiratory oncologic emergency, although there is relatively good prognosis.

## Background

Congenital mesoblastic nephroma (CMN), a rare benign renal stromal neoplasm, is the most common renal tumor in neonatal and early infancy periods [1]. It mainly presents as asymptomatic abdominal mass, but there have been some cases with hematuria [2], hypertension [3] and hypercalcemia [4]. Neonatal dyspnea early after birth due to rapid tumor growth is reported here for the first time. CMN was detected from the fetal period, and caused respiratory oncologic emergency after birth.

## Case presentation

A mother presented with abdominal distension at 32 weeks and 3 days of gestation. Ultrasonography (US) detected a 67 × 67 mm retroperitoneal tumor in the fetus and showed polyhydramnios. Fetal magnetic resonance imaging (MRI) two days later showed polyhydramnios and a 69 × 70 mm mass, low signal on T1-weighted imaging and faint high signal on T2-weighted imaging at the right kidney (Fig. 1). The mother presented worsening abdominal distention and signs of imminent preterm birth due to polyhydramnios. Maternal abdominal US at 34 weeks and 1 day of gestation showed the exacerbation of polyhydramnios and signs of imminent preterm birth. Amniocentesis was performed and the signs of imminent preterm birth were alleviated, but the renal tumor had increased to 80 × 100 mm at 35 weeks and 5 days of gestation. The management strategy for the fetus was scheduled cesarean section as early as possible and surgery for the renal tumor to avoid respiratory symptoms. Cesarean section was therefore performed at 36 weeks and 2 days of gestation. The birth weight was 2638 g and 1 and 5 min APGAR scores were 2 and 4 points, respectively. The neonate could not breathe spontaneously at birth and presented remarkable abdominal distension. After undergoing cardiopulmonary resuscitation, he entered our intensive care unit. Vital signs and physical findings at birth included a pulse rate of 169 bpm, SpO_2_ of 89%, blood pressure of 89/44 mmHg and body temperature of 36℃. He had a palpable mass on the right side of the abdomen. Blood tests at birth showed Hb of 9.5 mg/dL, and tumor markers such as HCGβ, AFP and NSE were within normal range. No occult blood was found on urinalysis at birth. Chest x-ray examination showed elevation of the diaphragm and compression of the thorax by renal tumor. Abdominal US showed a 79 × 98 mm tumor at the right kidney and exclusion of the liver to the cranial side. Abdominal computed tomography (CT) showed an 80 × 100 mm tumor that had an inhomogeneous contrast effect. The liver was excluded to the cranial side and the diaphragm was elevated by the renal tumor (Fig. 2).

**Fig. 1:** Fetal MRI at 32 weeks and 5 days of gestation. A 69 × 70 mm mass showing low signal on T1-weighted imaging and faint high signal on T2-weighted imaging was detected in the right kidney

**Fig. 2:** Chest and abdominal X-ray examination and contrast-enhanced CT at birth. Chest and abdominal X-ray showed elevation of the diaphragm and exclusion of the thorax. Contrast-enhanced CT showed an 80 × 100 mm mass in the right kidney that had an inhomogeneous contrast effect. The tumor excluded the liver to the cranial side and elevated the diaphragm

### Postnatal course

High-frequency oscillation ventilation and circulatory agonists were administered to maintain respiratory and circulatory systems. Arterial blood gas analysis used the following ventilation settings: FiO2 = 0.5, stroke volume = 30 mL and mean airway pressure = 16 mmHg. The pH was 7.286, PaCO_2_ was 49.0 mmHg, PaO_2_ was 142.0 mmHg, HCO_3_ was 23.4 mmol/L and BE was -3.4 mmol/L. Under the same ventilation settings at 1 day of age, there was suggestion of the progression of hypoxemia and respiratory acidosis (pH was 7.231, PaCO_2_ was 53.1 mmHg, PaO_2_ was 80.7 mmHg, HCO_3_ was 22.3 mmol/L and BE was -5.4 mmol/L). Emergency laparotomy was performed at one day after birth because exclusion of the diaphragm due to the right renal tumor may have been the cause of respiratory and circulatory insufficiency.

### Intraoperative findings

The liver and ascending colon were excluded by a dark red mass covering the peritoneum. The ascending colon was mobilized from the retroperitoneum and the tumor was detached from the surrounding tissue. The right renal artery and vein and the right ureter were dissected, and the right kidney was resected. The right adrenal gland was preserved.

### Findings of excised specimens and pathological findings

The tumor was covered with a capsule, and a yellow solid component and a renal parenchymal component were found on the cut surface (Fig. 3). The tumor contained normal renal tissue such as glomeruli and renal tubules. The perirenal adipose tissue had been invaded, but the surgical margin was negative. The tumor was composed of spindle-shaped cells, with a swollen oval-shaped nucleus. The number of mitotic figures was increasing and the tumor was intricate in a bundle. Immunohistochemical staining further showed negative WT-1, strong diffusely-positive α-SMA in cytoplasm, and partially-positive CD56 in cell membrane, which led to diagnosis of CMN (Fig. 4).

**Fig. 3:** Excised specimen findings. The tumor was macroscopically covered with a capsule. A yellow solid component including a normal renal parenchymal component was observed on the tumor cut surface

**Fig. 4:** Pathological findings. **A**: The tumor was histologically composed of spindle-shaped cells with an oval swollen nucleus and an increasing number of mitotic figures with a bundle.. HK collected data and wrote the manuscript. YM, TG and HY read and helped to write the manuscript. All authors read and approved the final manuscript. **B**, **C**, **D**: WT-1 was negative because the nucleus was not stained. α-SMA was diffusely strongly positive in cytoplasm (yellow arrow) and CD56 was partially positive in cell membrane (red arrow head) on immunological staining

### Postoperative course

Under arterial blood gas analysis (FiO2 = 0.4, f = 50/min, PIP = 18 mmHg and PEEP = 4 mmHg) the pH was 7.431, PaCO_2_ was 38.0 mmHg, PaO_2_ was 89.7 mmHg, HCO_3_ was 25.2 mmol/L and BE was 1.1 mmol/L. This suggested the improvement of hypoxemia and respiratory acidosis. Respiration and hemodynamics became stable after the operation. The circulatory agonist was discontinued on postoperative day (POD) 2 and the patient was extubated on POD 3. The postoperative course was uneventful, and the patient was discharged on POD 45. Thirty-six months have passed since the operation without adjuvant chemotherapy, and the infant has not had recurrence, metastasis or complications.

## Discussion and conclusions

CMN can often be diagnosed antenatally with US or MRI [5]. On US, characteristics of CMN include intra-tumoral hemorrhage, cysts and necrosis in well-defined solid tumors with hypoechoic regions. MRI shows low to equal signals on T1-weighted images and high signal on T2-weighted images compared with renal parenchyma as characteristics of CMN [6]. CMN and Wilms tumors exhibit similar characteristics on US and MRI, however, which makes it difficult to distinguish between them [7]. They are therefore often diagnosed by histopathological examination. On immunohistochemical staining, WT-1 staining is generally positive for Wilms tumors, but it is negative for CMN.

In the present case, US revealed a non-uniform hypoechoic region inside. MRI showed a low signal on the T1-weighted image and a faint high signal on the T2-weighted image. WT-1 was negative by immunohistochemical staining. US, MRI and immunostaining findings were consistent with CMN.

The earliest reported detection of CMN was at 22 weeks of gestation [8]. CMN is often detected as a fetal abdominal mass at around 30 weeks of gestation [9]. Approximately 70% of cases have polyhydramnios, which leads to a significantly higher risk of preterm birth and mothers may give birth due to fetal distress, perhaps prematurely [9]. CMN has also been reported to increase rapidly in size in late pregnancy [10], although the cause remains unknown. Strict and careful fetal management is therefore required during the perinatal period [11]. CMN with oligohydramnios was reported to have poor prognosis due to the difficulty of management [12], whereas CMN with polyhydramnios is sometimes managed by amniocentesis [13]. Leclair et al. reported a case in which emergency surgery was performed because of hemodynamic instability due to rupture of neonatal CMN [14]. Oncologic emergency associated with respiratory disorder, such as apnea or dyspnea due to CMN, has not been reported until now. In the present case, a renal tumor with polyhydramnios was detected at 32 weeks of gestation. Abdominal distension due to exacerbation of polyhydramnios and signs of imminent preterm birth were presented, and amniocentesis was performed. The signs of preterm birth were alleviated by amniocentesis, but the renal tumor gradually increased in size and led to exclusion of the thoracic cavity, which can cause postnatal respiratory distress. In this stage, it was thought that the fetus would not be under crucial respiratory distress immediately after birth because the fetus could be managed well without fetal distress after one-time amniocentesis, although tendency for increase in size of the renal tumor was noted. The management strategy was therefore cesarean section as early as possible and surgery for renal tumor before respiratory symptoms could be presented. The neonate was born by scheduled cesarean section at 36 weeks of gestation, presenting dyspnea and weak crying immediately after birth. The neonate could be resuscitated well because the possibility of respiratory dysfunction after birth. It was suggested, however, that ex utero intrapartum treatment (EXIT) should be indicated for not only huge cervical tumors or congenital high airway obstruction syndrome, but also lung tumors or diaphragmatic hernia that could cause remarkable dyspnea after birth [15]. There have been no reports on the effect of renal tumors upon the respiratory system in neonates or of EXIT for renal tumors. We suggest there should have been more discussion about indication for EXIT for the present fetus between members of pediatric surgery, pediatrics, gynecology and anesthesia departments. The renal tumor continued to increase in size after birth, and it reduced the volume of the abdominal and thoracic cavities, resulting in decreased diaphragmatic compliance. It was therefore thought that hypoxemia and respiratory acidosis progressed early after birth.

The standard treatment for CMN is surgical resection, and the 5-year survival rate is 93–96% [7]. Tumor rupture or incomplete tumor resection could, however, cause local recurrence or metastasis [16, 17]. In the present case, the tumor invaded the surrounding adipose tissue, and complete resection without rupture was performed. Histopathological examination showed negative surgical margin, so the rate of local recurrence or distant metastasis is therefore thought to be low.

In conclusion, neonates can have respiratory oncologic emergency because of a rapid increase in size of CMN that leads to dyspnea by elevation of the diaphragm and exclusion of the thorax, although CMN has a relatively good prognosis.

## Data Availability

Data sharing is not applicable to the present article as no datasets were generated or analyzed during the current study. All clinical data and images adopted in this article are contained in the medical records of Wakayama Medical University.

## Abbreviations

AFP: Alfa fetoprotein
BE: Base excess
CD56: Cluster of differentiation 56
CMN: Congenital mesoblastic nephroma
CT: Computed tomography
EXIT: Ex utero intrapartum treatment
FiO2: Fraction of inspiratory oxygen
HCGβ: Human chorionic gonadotropin beta subunit
HCO3: Hydrogen bicarbonate
MRI: Magnetic resonance imaging
NSE: Neuron-specific enolase
PaCO2: Partial pressure of arterial carbon dioxide
PaO2: Partial pressure of arterial oxygen
POD: Postoperative day
US: Ultrasonography
WT-1: Wilms' tumor gene 1
α-SMA: Alpha-smooth muscle actin
